# Examining Impacts of Acidic Bath Temperature on Nano-Synthesized Lead Selenide Thin Films for the Application of Solar Cells

**DOI:** 10.1155/2022/1003803

**Published:** 2022-01-11

**Authors:** Saka Abel, Jule Leta Tesfaye, N. Nagaprasad, R. Shanmugam, L. Priyanka Dwarampudi, Tyagi Deepak, Hongxia Zhang, Ramaswamy Krishnaraj, B. Stalin

**Affiliations:** ^1^Dambi Dollo University, College of Natural and Computational Science, Department of Physics, Dembidolo, Ethiopia; ^2^Centre for Excellence-Indigenous Knowledge, Innovative Technology Transfer and Entrepreneurship, Dambi Dollo University, Dembidolo, Ethiopia; ^3^Department of Mechanical Engineering, ULTRA College of Engineering and Technology, Madurai 625104, Tamilnadu, India; ^4^TIFAC CORE HD, Department of Pharmacognosy, JSS Academy of Higher Education and Research, Ooty, Tamilnadu, India; ^5^Department of Pharmacognosy, JSS Academy of Higher Education and Research, Ooty, Tamilnadu, India; ^6^Department of Management, Dambi Dollo University, Dembidolo, Ethiopia; ^7^State Key Laboratory of Biobased Materials and Green Paper Making, School of Food Science and Engineering, Qilu University of Technology, Shandong Academy of Sciences, Jinan, Shandong Province, China; ^8^Dambi Dollo University, College of Engineering and Technology, Department of Mechanical Engineering, Dembidolo, Ethiopia; ^9^Department of Mechanical Engineering, Anna University, Regional Campus Madurai, Madurai 625 019, Tamil Nadu, India

## Abstract

The influence of bath temperature on nano-manufactured PbSe (lead selenide) films was successfully generated by utilizing CBD on the acid solution's metal surface tool. Pb (NO_3_)_2_ was employed as a lead ion source as a precursor, while Na_2_O_4_Se was used as a selenide ion source. The XRD characterization revealed that the prepared samples are the property of crystalline structure (111), (101), (100), and (110) Miller indices. The scanning electron microscope indicated that the particles have a rock-like shape. There was a decrement of energy bandgap that is from 2.4 eV to 1.2 eV with increasing temperature 20°C–85°C. Thin films prepared at 85°C revealed the best polycrystal structure as well as homogeneously dispersed on the substrate at superior particle scales. The photoluminescence spectrophotometer witnessed that as the temperature of the solution bath increases from 20°C to 85°C, the average strength of PL emission of the film decreases. The maximum photoluminescence strength predominantly exists at high temperatures because of self-trapped exciton recombination, formed from O_2_ vacancy and particle size what we call defect centres, for the deposited thin films at 45°C and 85°C. Therefore, the finest solution temperature is 85°C.

## 1. Introduction

Currently, the world is in trouble with air and water pollution released from nonrenewable energy sources such as coal, natural gas, fossil fuels, and fabrics [1]. The fuels released from fabrics flow out to the rivers and cause water pollution. This polluted water is directly consumed by a person and cause diseases like cholera, amoebic dysentery, and typhoid. Generally, it harms human safety health in the world. Photovoltaic technology connects solar power renewable and sustainable energy. This renewable energy originates from natural assets that are continuously replaced. These include the sunlight, ocean, and the power of wind [2]. This technology of energy is deliberated unpolluted and does not contain carbon since it does not emit greenhouse gases [3]. Since it is a clean energy source, it has no influence on the atmosphere other than the energy coming from fossil coals. When they are burned, they release dangerous carbon toxic radiations into the environment [4]. To reduce these hazardous wastes and pollutions from the world, the production and fabrication of solar cells from compound semiconductor thin films is the only solution. Because currently, the existing elemental semiconductor is very expensive and anybody cannot use it [5]. A wide-ranging investigation has been dedicated to produce numerous kinds of semiconductor thin films which are applicable in renewable sources of energy like solar cells [6]. This is because of their potential uses in the production of photovoltaic materials, optical-electronic devices, and sensor and infrared indicator instruments [3]. The lead selenide thin films appeal consideration of many scholars because they involve low cost, exist in abundance, and retain semiconducting material goods [7].

The production of films like lead selenide has been discovered via so many methods. These include electrodeposition, CBD, electrochemical atomic layer, photochemical, and molecular beam epitaxial deposition method [6]. The films synthesized via solution techniques are generally inexpensive than films produced via the concentrated somatic methods. In the present work, the CBD technique was carefully chosen because of its many benefits like the inexpensive, wide scope of fabrication, and straightforwardness during the installation.

Present, chemical bath preparation techniques are used to synthesize many semiconductors films, including [8] zinc sulfide (ZnS), lead selenide (PbSe), cadmium selenite(CdSe), zinc selenite (ZnSe), Cu_2_S (copper sulphide), CuInS (copper indium sulfide), and CuBiS_2_ (copper bismuth sulfide) on glass substrates [9], and they have no longer quality.

There are very few chemically prepared PbSe films reported by using glasses substrates in an alkaline base. But this can make deletions of films and affect the quality of prepared films. Even they release toxic hydroxide chemicals during their depositions [10]. For the present work, we have used metallic substrates to grow lead selenide films via the CBD method in an acidic medium (pH = 4) for the applications of solar cells.

## 2. Instruments and Methodology

PbSe films were grown on a metallic substrate (30 × 70 × 1) mm by means of CBD techniques. Proceeding to preparations, the metal substrate was inserted in ethanol for about 15 min, tracked via ultra-sonically washed in deionized water again for 20 min, and lastly desiccated in warm condition. The solution of lead nitrate was used as a metallic precursor source that is lead, sodium selenite as the sulphide ion source, and [(HOC_2_H_4_)3N] as a complexing agent for synthesis of lead sulphide thin films [10, 11]. All compounds were analytically graded before the deposition, and the bath solutions were equipped with deionized seawater. Stepwise deposition, 25 ml of 0.2 M of lead nitrite was complexed with 15 ml of triethanolamine. Next, 15 ml of 0.2 M of sodium selenite was dropped step by step to the reaction. The pH values of the resultant solution were controlled by using droplet sulfuric acid [12] and then with continual stirring. The cleaned metal substrate was bought from a shop prepared to grow nanoparticles of lead selenide, with varying temperatures as 20°C, 45°C, and 85°C. As preparation time required, 95 min ended; we fetched the water from the chemical solution by using a syringe. The bottom of a glass of bath solution is left with molten lead selenide nanoparticles. Next, the metal substrates were coated with molten lead selenide, and it was dried in the air, splashed with deionized seawater and kept in an oven for further analysis.

Crystalline structures of nano-synthesized PbSe films were studied by using XRD, PANalytical, US [13]. The diffractometer is kept with CuK sources to operate at 35 kV and 23 *µ*A; the scanning was taken in a 2*θ* range from 20° to 85°. An optical absorption measurement was executed using a Janeway 6850 UV/visible spectrophotometer in the range of 226–2250 nm. The surface morphology study of nanoparticles size was characterized via scanning electron microscopy on a Hitachi SU5000 with an operating voltage of 20 kV. Photoluminescence of the prepared material was analyzed by using a photoluminescence spectrophotometer.

## 3. Results and Discussion

### 3.1. Structural Characterization

The X-rays diffraction patterns of the PbSe thin films deposited at different temperature bath solutions are shown in Figure 1. Thin films deposited at 45°C observed with four peaks at 2*θ* = 26°C and 30.6°C. When bath solution temperature rises to 85°C, the intensity of the peaks attributable to PbSe is revealed. The position of the peak along the (111), (101), (100), and (110) Miller indexes reveals the saturated intensity with well-defined sharp indicating high crystallinity of the material prepared. This means that the grain size of the grown thin film increases with the temperature of the bath. The number of peaks of PbSe films also increased when bath temperature increased. These witnesses show that the deposited structure has a cubic phase, matching with earlier reported data [12]. The three lattice constant values are equal to 6.13 Å. In this case, the presence of iron dioxide peaks in the XRD is because of the metallic substrate used to prepare films. The observed four peaks are at 2*θ* values, 40.2, 52.8, and 67.3. The peaks via solid triangles are related to the cubic shape of lead selenide, and those striking with undefended diamonds attributed to the orthorhombic crystal of iron dioxide. This result is witnessed with scanning electron microscope analysis homogeneous and cubic structure; this result agrees with a reported study [13]. Comparison of evaluated and standard “*d*” and 2*θ* values for nano-synthesized PbSe thin films with varying bath temperatures (20°C, 45°C, and 85°C) and deposition time 95 min is given in Table 1.

The size of the particle was premeditated by using Scherer's formula; it is given by

(1) $$\begin{array}{c} D=\frac{0.9\lambda }{\beta \;\cos\;\theta }, \end{array}$$

where *λ* shows the wavelength, *β* stands for the FWHM in rad, and *θ* represents the angle diffraction (Bragg angle).

From Table 1, it is possible to understand that the crystal size of the third sample is decreased at a higher temperature (at 85°C); this shows that when the temperature increases, the bonds between particles will break and the size becomes smaller and smaller.

### 3.2. Surface Morphology Characterization of PbSe Thin Films

The scanning electron microscope micrographs of PbSe thin films deposited at different temperatures are shown in Figure 2. Variation of temperatures shows a significant influence on the surface morphology of the thin films. All micrographs samples were taken at 10.00 kV and 20.71x magnification. Scanning electron microscopy reveals that lead selenide films grown at all temperatures fully covered the metal substrates. The synthesized films that had cracks were very small in size with well-covered grain borders. As the researcher, well-defined grains were observed for the film deposited at all temperatures, but the grains were decreasing with temperature increases from 20°C to 85°C. As it was observed in XRD analysis, the shape of PbSe films was cubic, and fully covered crystals on the metal substrate were investigated. Increasing temperature raises the smoothness of the films; the grain amounts were observed to rise slowly. Additionally, there is a material which just likes soil which was decreasing in size as shown in Figures 2(a)–2(c) with increasing bath temperature from 20°C to 85°C that shield over cadmium sulphide thin films in some amounts of the apparent. The impact of temperature on the surface morphology of nano-synthesized lead selenide films was observed; this is in good agreement with a reported study [14].

### 3.3. Optical Properties

The optical immersion of the nano-synthesized lead selenide films prepared from different temperatures was measured in the wavelength range of 226–2250 nm, which is in the visible region photocatalyst, as shown in Figure 3. The absorbance of the films expressively increased when the bath temperature increased within the deliberated range of wavelength. The highest absorption of thin films was witnessed in the visible wavelength (*λ*) range. The absorption coefficient of PbSe films was evaluated by using Lambert's equation:

(2) $$\begin{array}{c} \alpha =2.30\;\frac{A}{t}, \end{array}$$

where *A* is the absorbance, *α* is the absorption of coefficient, and *t* is stands for the thickness. The band gaps (*E*_*g*_) of films were calculated from Tauc's relation [15]:

(3) $$\begin{array}{c} {\left(\alpha hv\right)}^{n}=k\left(hv-E_{g}\right), \end{array}$$

where *h* is Planck's number, *v* stands for the frequency, *k* expresses the optical transition constant number, *E*_*g*_ is the energy of bandgap, and *n* is transition type, and it is varying either 2 or 2/3 for direct allowed and forbidden transitions or 1/2 or 1/3 for indirect allowed and forbidden transitions, correspondingly [16]. Best linear fit for equation (3) is given for *n* = 2 in the main absorption edge, representing that the thin films have direct optical band gaps. The (*αhv*) axis intercept attained by extrapolating the linear portion of the (*αhv*)^2^ vs. (*hv*) curve gives the *E*_*g*_ of the films as shown in Figure 3. The *E*_*g*_ of the nano-synthesized PbSe thin films declined from 2.4 eV to 1.2 eV with the temperature of the solution increasing from 20°C to 85°C. The bandgap decrement could be because of increment of crystal size with temperature; this result is the same as reported [17]. The maximum absorbance observed in visible light section and band gaps of thin films within the range of 2.6–1.2 eV in all PbSe thin films provides the application materials as the absorber layer in photovoltaic thin film solar cells as well as well-organized visible light photocatalyst [18–21].

### 3.4. Photoluminescence Property (PL)

Inappropriate to discover the optical study of deposited PbSe nanoparticles, photoluminescence was similarly used. In the *λ* range from 350 nm to 600 nm at different temperatures, the PL spectrum of nano-synthesized films was reported. When solution bath temperature increases from 20°C to 85°C, the average strength of PL decreases. The maximum photoluminescence strength is predominant because of the self-trapped exciton recombination, formed from O_2_ vacancy and particle size what we call defect centres, for the deposited thin films at 45°C and 85°C. The photoluminescence intensity rises sequentially with all temperatures.

Figure 4 shows the absorption of nano-synthesized lead selenide films deposited at various temperatures; all samples reveal a gradual rising absorbance in the visible area, which provides the potential for these tools to be applicable in a photovoltaic solar cell. The plotted figure shows that the samples synthesized at a greater temperature of the solution have greater absorption values related to other solution bath temperatures. Because these are nano-synthesized, thin films have the maximum uniform surface and well crystallinity compared with other reported samples.

## 4. Conclusions

Nano-synthesized lead selenide films are successfully prepared using an easy, inexpensive CBD technique in an acidic medium. Chemical solutions made from lead nitrate and sodium selenite compounds are to be sources of lead and selenide ions. The triethanolamine was served as a complexing mediator through the deposition procedure. The X-ray diffraction pattern tells the creation of a cubic crystalline structure with very tough peaks defined as (111), (101), (100), and (110) Miller indices plane. PL confirmed that photoluminescence emission of the deposited thin films increased with increasing bath temperature. The deposited film at 85°C indicated the best crystallite and is homogenously formed on a substrate with larger crystal sizes. Bandgap energy was declined from 2.4 eV to 1.2 eV with temperature increases from 20°C to 85°C, and this is suitable for photovoltaic solar cells.

## Figures and Tables

**Figure 1:** XRD plots of lead selenide films deposited at various bath temperatures: (a) 20°C. (b) 45°C. (c) 85°C.

**Figure 2:** The scanning electron microscope micrograph of nano-synthesized lead selenide films grown varying temperatures: (a) 20. (b) 45. (c) 85°C.

**Figure 3:** Plots of variation of optical absorption (*α*_*t*_) vs. wavelength films variation in bath temperature: (a) 20°C. (b) 45°C. (c) 85°C.

**Figure 4:** Photoluminescence spectra of nano-synthesized PbSe films grown at different temperatures: (a) 20°C. (b) 45°C. (c) 85°C.

**Table 1:** Comparison of evaluated and standard “*d*” and 2*θ* values for nano-synthesized PbSe thin films with varying bath temperatures (20°C, 45°C, and 85°C) and deposition time of 95 min.

Sample	Temperature (°C)	2*θ* (radians)	FWMH (°)	Crystal size (nm)
1	20	30.812	6.98	1.17
2	45	30.847	6.13	1.04
3	85	42.89	12.14	0.7

## Data Availability

The data used to support the findings of this study are included within the article.
